This article has been retracted.

# Implications of Human Antimicrobial Peptide Defensin Beta-1 in Clinical Oral Squamous Cell Carcinoma Patients via an Integrated Bioinformatics Approach

**DOI:** 10.1155/2022/2203615

**Published:** 2022-02-18

**Authors:** Simin Li, Hu Li, Yuzhen Xu, Wanchen Ning, Shaonan Hu, Shanzun Wei, Hongning Song, Jianghe Sun, Dirk Ziebolz, Gerhard Schmalz, Xianda Hu, Min Liu

**Affiliations:** ^1^Stomatological Hospital, Southern Medical University, Guangzhou 510280, China; ^2^Department of Rehabilitation, The Second Affiliated Hospital of Shandong First Medical University, Taian, Shandong Province 271000, China; ^3^Innovation Center Computer Assisted Surgery (ICCAS), Leipzig University, Semmelweisstraße 14, Leipzig 04103, Germany; ^4^Department of Urology, West China Hospital, Sichuan University, Chengdu 610000, China; ^5^Department of Stomatology, The Second Affiliated Hospital of Shandong First Medical University, Taian, Shandong Province 271000, China; ^6^Department of Cariology, Endodontology and Periodontology, University of Leipzig, 04103 Leipzig, Germany; ^7^Laboratory of Molecular Cell Biology, Beijing Tibetan Hospital, China Tibetology Research Center, 218 Anwaixiaoguanbeili Street, Chaoyang, Beijing 100029, China

## Abstract

**Background:**

The human antimicrobial peptide defensin beta 1 (DEFB1) has been found to play antimicrobial and anti-inflammatory roles in oral diseases; however, its tumor-regulating role in oral squamous cell carcinoma (OSCC) has not yet been researched by using an integrative bioinformatics approach.

**Objective:**

To investigate the regulating mechanisms of the DEFB1 gene in OSCC in terms of its expression patterns, prognostic values, biological functions, and implication for tumor immunity.

**Methods:**

The DEFB1 gene expression pattern and regulatory involvement in OSCC were investigated using publically accessible data from TCGA database. R software tools and public web servers were utilized to conduct statistical analysis of data from cancer and noncancerous samples.

**Results:**

DEFB1 was found to be significantly downregulated in OSCC tumor samples compared with healthy control oral samples. The DEFB1 gene was found associated with the prognostic outcomes of OSCC, and its upregulation represented better survival outcome. Gene set enrichment analysis (GSEA) results showed that DEFB1-significantly correlated genes were mainly enriched in four signaling pathways mediating the antitumor role of DEFB1 in OSCC, including extracellular matrix-related pathway, RTK/PI3K/AKT/mTOR pathway, keratinization, and cytokine-related pathway. The gene-gene interaction network showed that DEFB1 was closely correlated with several genes, for example, CCR6 (C-C motif chemokine receptor 6), CXCL1 (C-X-C motif chemokine ligand 1), MAP4K2 (mitogen-activated protein kinase kinase kinase kinase 2), PTGER3 (prostaglandin E receptor 3), and MMP7 (matrix metallopeptidase 7). Moreover, DEFB1 was found to be involved in the tumor immunity of OSCC by regulating the function of tumor macrophage cells, mast cells, T cells, and NK cells.

**Conclusions:**

Given the dysregulation, prognostic value, and tumor progression-related biological pathway alteration, indicating the tumor immune-modulatory role of DEFB1 in OSCC, the DEFB1 gene should be regarded as a potential therapeutic target for treating oral cancer.

## 1. Introduction

Antimicrobial peptides (AMPs) are short peptides with cationic charges, which are characterized by a broad spectrum of antibacterial activities and a low degree of resistance [1]. The cationic charges of AMPs allow AMPs to exhibit antibacterial activity by neutralizing lipopolysaccharide (LPS) [2]. In addition, AMPs are well-known because of their function in modulating the immune response and therefore are regarded as critical host defense molecules involved in human innate immunity [3]. Apart from their antibacterial and immune modulatory roles, AMPs have recently attracted considerable attention because of their regulating role in many cancers [4]. Defensins are part of the family of AMPs that are found in humans, and particularly, they have attracted great attention. Defensins are a family of small antimicrobial peptides with the size of 2–5 kDa and are characterized by a *β*-sheet core structure stabilized by three conserved intramolecular disulfide bonds [5]. Defensins consist of *α* and *β*-defensins in humans. Searching for oral cavity sourced AMPs in the Antimicrobial Peptide Database (APD) [6], several defensins were found to be sourced from the oral cavity, including neutrophil peptide-1 (HNP-1, encoded by DEFA1 gene), human neutrophil peptide-2 (HNP-2, encoded by DEFA1 gene), and human neutrophil peptide-3 (HNP-3, encoded by DEFA3 gene), as well as human beta-defensin 1 (hBD-1, encoded by DEFB1 gene), human beta-defensin 3 (hBD-3, encoded by DEFB103B gene), human beta-defensin 2 (hBD-2, encoded by DEFB4A gene), and human beta-defensin 114 (hBD-114, encoded by DEFB114 gene).

Previous research has reported that the expression patterns of defensin family genes in cancer vary depending on the type of defensin, as well as the type of cancer. Thus, a specific defensin might play either a promoting or inhibiting role in cancer progression [7]. Our primary research showed that among the six oral-sourced defensins, only the gene encoding DEFB1 was found to be dysregulated in oral squamous cell carcinoma (OSCC) based on TCGA-OSCC data. DEFB1 has been reported to be significantly downregulated in OSCC cell lines as compared with healthy gingival keratinocytes [8]. DEFB1 was found to play an antitumor role in OSCC by suppressing tumor migration and invasion; however, without influencing the proliferation or apoptosis of OSCC cells [9]. More importantly, DEFB1 expression has been shown as a prognostic indicator in OSCC [9]. However, the regulatory role of DEFB1 in OSCC tumor biology remains unclear. The concept of correlation between DEFB1 gene expression and clinical variables of OSCC is yet unknown. The signaling pathways through which DEFB1 could act in the pathogenesis of OSCC, as well as its role in tumor immunity of OSCC, need to be further investigated. To the authors' knowledge, there is no report using a systematic approach to investigate putative regulating mechanisms of the DEFB1 gene involvement in OSCC. Therefore, the potential biological mechanisms in DEFB1-mediated regulation of OSCC were selected as the focus of the present study.

## 2. Materials and Methods

### 2.1. Procurement of Oral-Sourced Defensin Family Antimicrobial Peptide Genes

The human oral cavity-sourced antimicrobial peptides (ADMs) were obtained from the Antimicrobial Peptide Database (APD, URL: https://aps.unmc.edu/database/anti) [6]. The AMP Database was searched with the source organism defined as oral/saliva/salivary gland/tongue/gingiva; 24 AMPs were obtained. The APD ID, source, and encoded genes of these ADMs are shown in Table 1. Among these oral-sourced AMPs, six defensin genes (DEFA1, DEFA3, DEFB103B, DEFB4A, DEFB1, and DEFB114) were identified to encode defensin family antimicrobial peptides; for example, DEFA1 encodes human neutrophil peptide-1 (HNP-1) and human neutrophil peptide-2 (HNP-2); DEFA3 encodes human neutrophil peptide-3 (HNP-3); DEFB103B encodes human beta defensin 3 (hBD-3); DEFB4A encodes human beta defensin 2 (hBD-2); DEFB1 encodes hBD-1 (human beta-defensin 1); and DEFB114 encodes human beta defensin 114.

### 2.2. The Aberrant Expression of Six Defensin Family Genes in OSCC Based on TCGA Data

Level 3 HT-seq data of head and neck squamous cell carcinoma (HNSC) patients with the FPKM format were downloaded from TCGA database. The samples without clinical information were removed. The OSCC samples with the anatomic sites of alveolar ridge, base of tongue, buccal mucosa, floor of mouth, hard palate, oral cavity, and oral tongue were retained, while the samples with the anatomic sites of hypopharynx, larynx, lip, oropharynx, and tonsil were removed. Thereby, 361 samples containing 329 OSCC tumor samples and 32 healthy control samples were included for the subsequent analysis based on TCGA-OSCC data. In brief, RNA-seq data with FPKM (Fragments Per Kilobase per Million) format was normalized into TPM (transcripts per million reads) format and then log2 transformed. The mRNA expression of six defensin family ADM genes (i.e., DEFA1, DEFA3, DEFB103B, DEFB4A, DEFB1, and DEFB114) in OSCC was analyzed and visualized by using the ggplot2 package (version 3.3.3) in R program (version 3.6.3). Unpaired and paired sample analyses were both performed. For the paired sample analysis, if the samples satisfied the Shapiro-Wilk normality test (*p* > 0.05), a paired sample *t* test was used. For the unpaired sample analysis, as the samples did not satisfy the normality test (*p* < 0.05), the Mann–Whitney *U* test (also named Wilcoxon rank sum test) was used. The results of this preliminary research showed that among these six defensin-family ADM genes, only DEFB1 was found to be significantly dysregulated in OSCC tumor tissues compared to healthy control oral tissues, while the other five defensin genes (i.e., DEFA1, DEFA3, DEFB103B, DEFB4A, and DEFB114) were not differentially expressed in OSCC tissues. Based on these findings, the DEFB1 gene was used as the research focus of the present study.

### 2.3. The Aberrant Expression of DEFB1 in Pancancer Data including HNSC

The mRNA expression levels of DEFB1 in multiple cancers including HNSC were analyzed and visualized by using the ggplot2 package (version 3.3.3) in R program (version 3.6.3). 15,776 samples' RNA-seq data from TCGA and GTEx in TPM (transcript per million) format was downloaded from UCSC XENA (URL: https://xenabrowser.net/datapages/), which had been uniformly processed by the Toil process [10]. Transcript mapped data were normalized to TPM format and then log2 transformed. The Mann–Whitney *U* test (also called the Mann–Whitney Wilcoxon test or the Wilcoxon rank sum test) was used for comparing the difference in DEFB1 mRNA expression between two groups (i.e., healthy control group and tumor group).

### 2.4. DNA Methylation Analysis of DEFB1 Gene in OSCC

Since MethSurv webserver for analyzing DNA methylation data only contained HNSC TCGA data instead of OSCC data [11], the potential association between DEFB1 DNA methylation and the pathogenesis of OSCC in the TCGA project was analyzed by using R program (version 3.6.3) and visualized using ggplot2 package (version 3.3.3). The analysis was based on the Illumina human methylation 450 data with beta format and contained 379 TCGA-OSCC tumor samples. The methylation data matched with 343 OSCC samples' RNA-seq data. The statistical analysis included the Shapiro-Wilk normality test, and Pearson correlation test was applied. The correlation between DEFB1 and each of the six methylation sites (e.g., cg20710667, cg02465761, cg24292612, cg01691696, cg19033555, and cg10076006) was investigated.

### 2.5. Procurement of Clinical Information of TCGA-OSCC Data Set

The subsequent analysis was based on TCGA-OSCC data set obtained in the previous step. The expression levels of DEFB1 mRNA, clinicopathological details, and general information of OSCC were obtained. The categorical variables included TNM stage (T stage, N stage, and M stage), clinical stage, primary therapy outcome, radiation therapy, gender, race, age, smoker, alcohol history, histologic grade, anatomic neoplasm subdivision, lymphovascular invasion, lymph node neck dissection, OS event, DSS event, and PFI event. If all levels of a certain categorical variable satisfied the conditions of theoretical frequency > 5 and total sample size > 40, the chi-square test was used. However, if any level in a certain categorical variable did not satisfy the condition of theoretical frequency > 5 and total sample size > 40, Fisher's exact test was used. If the data of a certain categorical variable were not normally distributed (*p* < 0.05), the Wilcoxon rank sum test was used. The analysis was performed in R program (version 3.6.3). OSCC samples were divided into two groups with a cutoff set as the median value of DEFB1 expression. Correspondingly, frequencies of the categorical variable levels in the low versus high-expression group of the DEFB1 gene were determined.

### 2.6. The Relationship between Clinical Characteristics and DEFB1 Expression

DEFB1 mRNA expression was observed in groups based on 17 types of clinical variables, e.g., T stage, N stage, M stage, clinical stage, radiation therapy, primary therapy outcome, gender, race, age, histological grade, anatomic neoplasm subdivision, smoker, alcohol history, lymph node neck dissection, OS event, DSS event, and PFI event. If the data for a certain clinical variable was normally distributed (*p* > 0.05), the Shapiro-Wilk normality test was used; otherwise, the Kruskal-Wallis test was used. The statistical analyses were performed and visualized by using the ggplot2 package in R program and included the 329 OSCC tumor samples.

In addition, the relationships between DEFB1 expression levels and clinical features were also investigated by using a binary logistics model. The independent variable—DEFB1—was divided into two categories, low expression and high expression of DEFB1, where the low expression of DEFB1 was used as the reference level. The dependent variable characteristics were also divided into two different categories, including T stage (higher T stage (T3 and T4) vs. lower T stage (T1 and T2)); N stage (presence of cancer spread to nearby lymph nodes (N1 and N2 and N3) vs. absence of cancer spread to nearby lymph nodes (N0)); M stage (M1 (presence of metastasis) vs. M0 (without metastasis)); clinical stage (higher clinical stages (Stage III and Stage IV) vs. lower clinical stages (Stage I and Stage II)); histologic grade (higher histologic grade (G3 and G4) vs. lower histologic grade (G1 and G2)); gender (male vs. female); race (Asian and Black or African American vs. White); age (>60 vs. ≤60); smoker (yes vs. no); alcohol history (yes vs. no); primary therapy outcome (PD and SD vs. PR and CR); radiation therapy (no vs. yes); lymph node neck dissection (yes vs. no); and lymphovascular invasion (yes vs. no). For each of these, the latter levels were considered as the reference.

### 2.7. Survival Analyses to Investigate the Prognostic Value of DEFB1 in Pancancer

The Gene Expression Profiling Interactive Analysis 2 (GEPIA2) (http://gepia.cancer-pku.cn/index.html) is an online database that consists of 9736 tumors and 8587 normal samples from TCGA and GTEx data [12]. Given a list of custom cancer types, GEPIA2 can provide a survival heat map depicting survival analysis results of gene lists based on multiple cancer types and was utilized. In the survival map, red blocks indicate that the increased expression of genes predicts worse prognosis and higher risk of death, and blue blocks represent that the increased expression of genes predicts better prognosis and lower risk of death. The blocks with darkened frames indicate statistical significance in prognostic analyses. Two types of prognostic outcomes (i.e., OS (overall survival) and DFS (disease-free survival)) were selected and analyzed in the survival map. “DEFB1” was used as the input of “Single Gene Analysis” module, and the survival analysis was performed to investigate the prognostic values of DEFB1 gene in pancancer by using a survival map with months as the survival time unit. Cutoff-high (50%) and cutoff-low (50%) values were used as the expression thresholds for splitting the high-expression and low-expression cohorts; and *p* value (no adjustment) < 0.05 was set as the significance level.

### 2.8. Survival Analyses to Investigate the Prognostic Value of DEFB1 in OSCC

Within TCGA-OSCC data set, only tumor samples with survival information were used for the survival analysis. Kaplan-Meier analysis was performed to compare the survival rate between the high and low DEFB1 gene expression groups using the *p* value determined in the log-rank test. The statistical analysis was done using the survival package (version 3.2-10) in R, and the Kaplan Meier (KM) plots were visualized by the survminer package (version 0.4.9) in R. Cox regression was used as the statistical analysis, and tumor samples were divided into groups according to the expression level of DEFB1: the low expression group of DEFB1 and the high-expression group of DEFB1. Three types of prognostic parameters were analyzed including overall survival (OS), disease-specific survival (PSF), and progress-free interval (PFI).

### 2.9. Subgroup Survival Analyses

Subgroup survival analysis was performed in order to investigate if DEFB1 mRNA overexpression can significantly affect the overall survival outcome of OSCC tumor cases belonging to specific subgroups based on the clinical characteristics including T stage, N stage, M stage, clinical stage, radiation therapy, primary therapy outcome, gender, race, age, histologic grade, anatomic neoplasm subdivision, smoker, alcohol history, lymphovascular invasion, and lymph node neck dissection. For the subgroup survival analysis, only one prognostic parameter was selected, which was overall survival (OS). Cox regression was used as statistical analysis. Statistical analysis of the survival information was analyzed by using the survival package (version 3.2-10) in R, and the Kaplan Meier (KM) plots were visualized by the survminer package (version 0.4.9) in R.

### 2.10. Survival Analysis by Univariate and Multivariate Cox Regression

The association between clinical variables and prognosis was investigated by performing univariate and multivariate Cox regression analyses. The coxph function in the survival package (version 3.2-10) of R program (version 3.6.3) was applied, and cox regression module was used in the statistical analyses. The prognostic type was selected to be overall survival. The clinical variables included in this analysis consisted of T stage, N stage, M stage, age, gender, race, smoker, clinical stage, alcohol history, histologic grade, radiation therapy, primary therapy outcome, lymphovascular invasion, lymph node neck dissection, anatomic neoplasm subdivision, and DEFB1 expression. During the process of variable grouping, lower T stage (T1 and T2), N stage (N0), M stage (M0), age (≤60 years old), gender (female), race (White), smoker (No), lower clinical stage (Stage I and Stage II), alcohol history (no), histologic grade (G1 and G2), radiation therapy (yes), primary therapy (PR and CR), lymphovascular invasion (no), lymph node neck dissection (yes), anatomic neoplasm subdivision (oral tongue), and DEFB1 expression (expression level of higher than median value) were used as the reference group.

### 2.11. Forest Plots

According to the results (HR, 95% CI, *p* value) obtained by univariate and multivariate cox regression analysis, two forest plots were plotted by using the ggplot2 package (version 3.3.3) in the R program (version 3.6.3). Every HR (hazard ratio) represents a relative risk of death that compares one instance of a binary feature to the other instance—reference. An HR > 1 indicates an increased risk of death, while an HR < 1 represents a decreased risk of death.

### 2.12. Nomogram Plotting

A predictive nomogram for OSCC by combining the expression values of DEFB1 with clinical variables has not been reported. Therefore, we constructed a prognostic nomogram by integrating clinical factors and gene expression using TCGA-OSCC data set. The nomogram was plotted by using the rms package (version 6.2-0) and survival package (version 3.2-10) in R program (version 3.6.3) and by following the Cox regression statistical analysis. Overall survival (OS) was chosen as the prognostic type. The included variables were T stage, N stage, M stage, clinical stage, histologic stage, age, race, gender, smoker, alcohol history, radiation therapy, primary therapy outcome, lymph node neck dissection, and lymphovascular invasion, as well as the expression of DEFB1.

### 2.13. Calibration Plot

The calibration plots were generated by using the rms package (version 6.2-0) and survival package (version 3.2-10). In the calibration plot, the fit between the actual observed fraction survival probability and the nomogram model-predicted survival probability under three time points (1-year, 3-year, and 5-year) was plotted in order to evaluate the prediction accuracy of nomogram model on predicting the actual prognostic results. If the solid lines regarding 1-year, 3-year, and 5-year fit the 45-degree ideal diagonal line very well, then it was indicated that the nomogram model achieved the perfect prediction.

### 2.14. ROC Curves to Evaluate the Diagnostic Value of DEFB1 mRNA Expression in OSCC

ROC curve analysis of DEFB1 gene expression data was conducted by using the pROC package (version 1.17.0.1) and visualized by ggplot2 package (version 3.3.3) in the R program (version 3.6.3). The predicated outcome parameters included clinical status (OSCC tumor vs. normal); T stage (T3 and T4 vs. T1 and T2); N stage (N1 and N2 and N3 vs. N0); clinical stage (Stage III and Stage IV vs. Stage I and Stage II); histologic grade (G3 and G4 vs. G1 and G2); gender (male vs. female); race (Asian and Black or African American vs. White); age (>60 vs. ≤60); smoker (yes vs. no); alcohol history (yes vs. no); anatomic neoplasm (alveolar ridge and base of tongue and buccal mucosa and floor of mouth and hard palate and oral cavity vs. oral tongue); primary therapy outcome (PD and SD vs. PR and CR); radiation therapy (no. vs. yes); lymphovascular invasion (yes vs. no); lymph node neck dissection (no vs. yes); OS event (dead vs. alive); DSS event (dead vs. alive); PFI event (dead vs. alive). In the ROC curves, the *x*-axis represents the false-positive rate (FPR), and the *y*-axis represents the true-positive rate (TPR). The area under the ROC curve (AUC) with an area greater than 0.9 indicates high accuracy; while 0.7-0.9 indicates moderate accuracy, 0.5-0.7 indicates low accuracy, and 0.5 indicates a chance result. The AUC and confidence interval (CI) corresponding to the all predicted outcomes were listed in the table format. The ROC curves of the predicated outcome with AUC of greater than 0.7 were presented, while the ROC curves of the other predicted outcomes with AUC of less than 0.7 were not presented.

### 2.15. Construction of Protein-Protein Interaction (PPI) Network

A protein-protein interaction (PPI) network of DEFB1 coexpressed genes was constructed using the STRING (https://string-db.org) database (version 11.5). The advanced setting was defined as follows: (1) network type: full STRING network; (2) required score: high confidence (0.700); and (3) size cutoff: no more than 20 interactors. The TSV file of the obtained PPI network was imported into Cytoscape software (version 3.8.2), and then, the NetworkAnalyzer tool was used for analyzing the network. The genes with a degree of greater than 10 were defined as hub genes. The top 10 genes with the greatest degree were obtained, and also, these 10 genes' correlation coefficients (*r*, “cor_pearson” value) were also obtained and summarized in a table.

### 2.16. Construction of Gene-Gene Interaction (GGI) Network

The GeneMANIA webserver (URL: http://genemania.org) was used for constructing the DEFB1-based gene-gene interaction network (GGI). The DEFB1 gene was used as the input, and top several functions with the smallest FDR value were selected in the network. The network consisted of DEFB1 and its 20 correlated genes. The GGI network was constructed by the automatically selected weighting method; after then, the network image and report were saved.

### 2.17. Identification of the Significantly Correlated Genes of DEFB1 in OSCC

The correlation analysis of a single gene-DEFB1 was performed by using the stat package (version 3.6.3) in R (version 3.6.3). The Pearson correlation test, as a parameter correlation test, can measure whether there is a linear relationship between the two groups and was used as the statistical analysis. After performing such analysis, only protein coding genes were retained. The cor_pearson value is the Pearson correlation coefficient “*r*” and obtained by Pearson analysis method. Generally, a cor_pearson value of greater than 0.7 is considered a strong correlation; a cor_pearson value between 0.5 and 0.7 indicates a moderate correlation, while a cor_pearson value of less than 0.4 is considered a weak or no correlation. Based on this rule, genes with ∣cor_pearson | >0.4 and *p*_pearson < 0.001 were defined as significantly correlated genes. The positive value of cor_pearson represents a positive correlation between DEFB1 and a certain gene, while the negative value of cor_pearson represents the negative correlation between DEFB1 and a certain gene.

### 2.18. Heatmap Plotting of DEFB1 Top 20 Correlated Genes

After defining the significantly correlated genes of DEFB1, the top 10 genes' list ranked by the descending order of the cor_pearson value was obtained and regarded as the top 10 positively correlated genes of DEFB1, while the top 10 genes' list ranked by the ascending order of the cor_pearson value was obtained and regarded as the top 10 negatively correlated genes of DEFB1. A heat map was plotted to show the expression pattern of these 20 correlated genes in OSCC samples. The heat map was visualized by using the ggplot2 (version 3.3.3) in R program (version 3.6.3).

### 2.19. Functional Enrichment Analysis of Significantly Correlated Genes of DEFB1

The genes with ∣cor_pearson | >0.4 and *p*_pearson < 0.001 identified previously were used for the functional enrichment analysis and gene set enrichment analysis to identify the significantly enriched functional terms of DEFB1-correlated genes. The gene names were converted to the Entrez ID by using the org.Hs.eg.db package (version 3.10.0) in R program (version 3.6.3). The functional enrichment analysis was performed using the clusterProfiler package (version 3.14.3) in R program (version 3.6.3). The species for the analysis was selected as Homo sapiens. The Benjamini and Hochberg (BH) method was used for calculating the adjusted *p* values. The GO terms including BP (biological process), CC (cellular component), and MF (molecular function) and KEGG pathways that were significantly enriched by the correlated genes were identified by setting the threshold of *p*.adj < 0.05 and *q* value < 0.2. If there were more than 30 terms which were significantly enriched by this threshold setting, then only the top 30 terms ranked by the ascending order of the *p* adjustment value were obtained to plot the bubble chart; otherwise, all of the terms were used for plotting the bubble chart. The bubble charts were plotted to visualize the enrichment results by using the ggplot2 package (version 3.3.3) in R program (version 3.6.3).

### 2.20. GSEA

The differentially expressed genes (DEGs) dysregulated between OSCC samples and healthy control samples were identified by using the DESeq2 (version 1.26.0) in R program (version 3.6.3) and based on TCGA-OSCC data set [13]. When performing the differential expression analysis, the experimental group was established as clinical status-tumor samples, while the reference group was established as clinical status-healthy control samples. The log2FC (fold change) value of the DEFB1-significantly correlated genes was obtained and used for the gene set enrichment analysis (GSEA). GSEA [14] was performed by using the clusterProfiler package (version 3.14.3) in R program (version 3.6.3) [15]. The pathways were obtained by three databases including KEGG pathway database, WikiPathways (WP) database, and Reactome (REAC) database. The referenced gene set was c2.cp.v7.2.symbols.gmt (Curated) in the MSigDB Collections (URL: https://www.gsea-msigdb.org/gsea/msigdb/collections.jsp#C2). The functional terms satisfying the condition of *p*.adjust < 0.05, false discovery rate (FDR) (also named *q* val) < 0.25 and ∣NES | >1 were considered as significantly enriched terms.

### 2.21. The Correlation between DEFB1 Expression and Immune Cells in OSCC

The correlation between the DEFB1 gene and immune cells in OSCC tumor samples was investigated by using the Pearson statistical method. Such analysis was performed by using the GSVA package (version 1.34.0) in R program (version 3.6.3) [16]. The ssGSEA algorithm, as a built-in algorithm in the GSVA package, was used in the statistical analysis. The analyzed 24 tumor immune infiltration cells (TIICs) consisted of aDC (activated DC), B cells, CD8 T cells, cytotoxic cells, DC, eosinophils, iDC (immature DC), macrophages, mast cells, neutrophils, NK CD56bright cells, NK CD56dim cells, NK cells, pDC (Plasmacytoid DC), T cells, T helper cells, Tcm (T central memory), Tem (T effector memory), Tfh (T follicular helper), Tgd (T gamma delta), Th1 cells, Th17 cells, Th2 cells, and Treg cells. The genetic markers of 24 TIICs were obtained from a paper authored by Prof. Bindea et al. [17]. Lollipop plot was used for illustrating the correlation between DEFB1 expression and 24 TIICs in OSCC samples. For the specific type of immune cell with statistical significance, scatter plots were used to show the correlation between DEFB1 expression and this specific type of cell in OSCC samples.

### 2.22. The Correlation between DEFB1 and 15 Classic Immune Checkpoint Genes (ICGs)

The 15 immune checkpoint genes (ICGs) were selected from a systematic review of ICGs in cancer [18, 19], including CD274, CTLA4, LAG3, HAVCR2, TIGIT, VSIR, CD276, VTCN1, BTLA, IDO1, CD70, CD40, CD47, TNFRSF18, and TNFSF14. The correlation between DEFB1 expression and any one ICG's expression in OSCC was evaluated by using the Pearson statistical method. The correlation coefficient *r* < 0 and *p* value < 0.05 represent significantly negative correlation, and conversely, a correlation coefficient *r* > 0 and *p* value < 0.05 represented significantly positive correlation in OSCC. A heat map was plotted to show the expression pattern of 15 ICGs in OSCC tumor samples. For the ICGs that were found to be statistically significant in the correlation with DEFB1, scatter plots were used to show the correlation between DEFB1 and each of these ICGs. Both the heat map and scatter plots were visualized by using the ggplot2 package (version 3.3.3) in R program (version 3.6.3).

## 3. Results

### 3.1. Flowchart of the Current Study

The study design of the current research followed was aligned with that of similar studies that investigated the involvement of a particular gene in a specific cancer [20–26].  Figure 1 presents a flowchart to visualize the study design of the current research. In the 1^st^ step, TCGA-OSCC data including 329 OSCC tumor samples and 32 healthy control samples were procured. In the 2^nd^ step, unpaired and paired sample analyses were performed to investigate the expression pattern of the DEFB1 gene in pancancer and OSCC. In the 3^rd^ step, the correlation between the DEFB1 gene and six DNA methylation sites was investigated by scatter plots. In the 4th step, survival analysis was performed to investigate the prognostic values of DEFB1 in pancancer and OSCC; and univariate and multivariate cox regression analysis was also performed. In the 5^th^ step, logistic regression analysis was performed to investigate the relationship between the DEFB1 gene and various clinicopathological variables. In the 6^th^ step, the gene-gene interaction (GGI) network and protein-protein interaction (PPI) network were constructed. In the 7^th^ step, the receiver operating characteristic (ROC) analysis was performed to evaluate the diagnostic accuracy of DEFB1 in various clinicopathological variables. In the 8^th^ step, gene correlation analysis was performed to explore the significantly correlated genes; and these genes' involved biological functions were explored by performing functional enrichment analysis and gene set enrichment analysis (GSEA). In the 9^th^ step, the involvement of DEFB1 in tumor immunity was investigated from the aspect of its correlation with 22 types of tumor-infiltrating immune cells and 15 typical immune checkpoint genes.

### 3.2. The Expression Pattern of Six Defensin Family Genes in OSCC

Figures 2(a) and 2(b) show that the median expression level of three defensin genes (DEFA1, DEFA3, and DEFB103B) in either OSCC tumor tissues or healthy control oral tissues was almost zero. The expression levels of DEFB4A in OSCC tumor tissues were higher than those in healthy control oral tissue, however, without showing statistically significant difference. Among these six defensin genes, only the DEFB1 gene was found to be dysregulated in OSCC tumor tissues compared with healthy control oral tissues.

### 3.3. The Expression Pattern of DEFB1 Gene in OSCC

The results of unpaired sample analysis (Figure 2(c)) and paired sample analysis (Figure 2(d)) were consistent, showing that only the DEFB1 gene was significantly downregulated in OSCC samples compared with healthy control oral samples. Figure 2(c) used the Mann–Whitney *U* test based on 329 OSCC tumor samples and 32 healthy control samples, and the expression of DEFB1 was lower in OSCC samples than that in healthy control samples, and the median difference between the two groups was -1.643 (-2.305−-1), with statistically significant difference (*p* < 0.001). Figure 2(d) used paired sample *t* test based on 32 OSCC tumor samples and their 32 paired healthy control samples and showed that the expression of DEFB1 in OSCC tumor samples was lower than that in healthy control samples, and the median difference between the two groups was -2.042 (-2.83−-1.253), with statistically significant difference (*t* = −5.282, *p* < 0.001).

### 3.4. Dysregulation of DEFB1 in Pancancer

The transcription level of the DEFB1 gene in pancancer was evaluated by analyzing TCGA RNA-seq data and is shown in Figures 2(e) and 2(f). DEFB1 mRNA expression was remarkably lower in HNSC tissue compared with normal head and neck tissue. Apart from its low expression in HNSC, DEFB1 was also found to be statistically significantly downregulated in several other cancers, for example, ACC, BRCA, GBM, KIRC, KIRP, LGG, PAAD, PRAD, and SKCM. However, DEFB1 was found to be statistically significantly upregulated in several cancers, for example, CHOL, ESCA, KICH, LAML, LUAD, LUSC, OV, READ, TGCT, THCA, THYM, UCEC, and UCS. In several cancers DEFB1 was not aberrantly expressed including BLCA, CESC, COAD, DLBC, LIHC, PCPG, and STAD.

### 3.5. Correlation between DEFB1 Gene and DNA Methylation Sites

DNA methylation analysis of six methylated sites revealed that two sites (cg19033555 and cg10076006) contained too many missing values after matching sample Ids. These two methylated sites could not be analyzed, since it was found that the effective samples of these two probes were less than 5. The correlation between the DEFB1 gene and the other four sites (e.g., cg20710667, cg02465761, cg24292612, and cg01691696) is visualized in Figure 2(g). A significant positive correlation was observed between methylation site-cg20710667 and the expression level of DEFB1 (Pearson correlation coefficient *r* value = 0.290, *p* < 0.001). A significant negative correlation was observed between methylation site-cg01691696 and the expression level of DEFB1 (Pearson correlation coefficient *r* value = −0.160, *p* = 0.003). The other two methylation sites (i.e., cg02465761 and cg24292612) were not found to be significantly correlated with the expression level of DEFB1 (cg02465761: *r* = 0.047, *p* = 0.392; cg24292612: *r* = −0.025, *p* = 0.65).

### 3.6. Clinical Characteristics of TCGA-OSCC Patients

The clinical and gene expression data of 329 primary OSCC tumor samples were downloaded from TCGA database (Table 2). Table 2 shows that only two clinical variables (i.e., histological grade and alcohol history) were statistically significantly related to the expression of the DEFB1 gene (*p* value < 0.05); however, the relationships with any of the other 16 clinical variables (i.e., TNM stage (T stage, N stage, M stage), clinical stage, primary therapy outcome, radiation therapy, gender, race, age, smoker, anatomic neoplasm subdivision, lymphovascular invasion, lymph node neck dissection, OS event, DSS event, and PFI event) and DEFB1 expression were not found to be statistically significant (*p* > 0.05).

### 3.7. Identification of the Clinical Variables Which Were Significantly Related to DEFB1 Expression

Among 17 clinical characteristics, only four clinical variables (i.e., histological grade, lymph node neck dissection, alcohol history, and OS event) were found to be statistically significantly related to the expression level of the DEFB1 gene (Figure 2(h)); while the other 13 clinical variables were not found to be significantly related to the expression of the DEFB1 gene. The DEFB1 mRNA expression levels of OSCC patients with higher histologic grade G3 were lower than those of patients with lower histological grade G1 (*p* = 0.036). DEFB1 mRNA expression levels of OSCC patients with lymph node neck dissection were higher than those of patients without lymph node neck dissection (*p* = 0.014). DEFB1 mRNA expression levels of OSCC patients with alcohol history were lower than those of patients without alcohol history (*p* = 0.006). DEFB1 mRNA expression of alive OSCC patients was higher than that of dead OSCC patients (*p* = 0.035).

Table 3 presents the results of logistic analysis and shows the association between DEFB1 expression and clinical features in patients with OSCC. Each row in the table represents a binary logistic regression model. The independent variable is the gene, DEFB1, and the low expression of DEFB1 is used as the reference; the dependent variable is the clinical characteristic, and the characteristic at the right side vs. that in brackets is the reference level of the dependent variable. Table 3 shows that the mRNA expression of DEFB1 was significantly associated with alcohol history (yes vs. no: OR = 0.532, 95% confidence interval (CI) = 0.329-0.853, *p* = 0.009); however, the mRNA expression of DEFB1 was not significantly associated with the other clinical variables.

### 3.8. Results of Survival Analyses of DEFB1 in Pancancer and Particularly OSCC

Figures 3(a) and 3(b) present the survival heat maps of hazard ratio (HR) to show the prognostic impacts of the DEFB1 gene on the overall survival (OS) and disease-free survival (DFS) outcomes of multiple cancer types, which were visualized based on the GEPIA2 database. When considering the overall survival, high expression of DEFB1 indicated worse prognosis in lung adenocarcinoma (LUAD) and pancreatic adenocarcinoma (PAAD), while the high expression of DEFB1 indicated improved prognosis in HNSC. When considering the disease-free survival, the high expression of DEFB1 indicated worse prognosis in cholangiocarcinoma (CHOL).

Figure 3(c) using the survival map showed the prognostic values of the DEFB1 gene in OSCC, in terms of three prognostic types (overall survival, disease-specific survival, and progress-free interval). Based on the fact that OSCC comprises the major type of HNSC, the prognostic results obtained in OSCC should be consistent with the results obtained in HNSC and accordingly, the difference of overall survival time distribution was statistically significant between the low- and high-expression groups of DEFB1 (*p* = 0.039), indicating that the high-expression group of DEFB1 was associated with better overall survival outcome. There was no statistical difference in disease-specific survival time distribution between two groups (*p* = 0.134), indicating that the expression of DEFB1 was not associated with the disease-specific survival outcome. The difference of progress-free interval time distribution between the low- and high-expression groups of DEFB1 (*p* = 0.049) was statistically significant, indicating that the high-expression group of DEFB1 was associated with better progress-free interval outcome.

### 3.9. Results of Subgroup Survival Analyses

Subgroup survival analysis indicated that DEFB1 mRNA overexpression significantly affected the overall survival outcome of OSCC tumor cases belonging to the subgroup of higher T stage T3/T4 (*p* = 0.046), M0 (*p* = 0.033), female (*p* = 0.036), age of >60 years old (*p* = 0.005), being smoker (*p* = 0.026), without having received radiation therapy (*p* = 0.005), primary therapy outcome showing PR and CR (*p* = 0.001), without lymphovascular invasion (*p* = 0.005), and with lymph node neck dissection (*p* = 0.026), respectively (Figure 3(d)).

However, DEFB1 mRNA overexpression did not significantly affect the overall survival outcome of OSCC tumor cases belonging to the subgroup of T1/T2 (*p* = 0.239), N0 (*p* = 0.056), N1 and N2 and N3 (*p* = 0.329), clinical stages I and II (*p* = 0.379), clinical stages III and IV (*p* = 0.1), having received radiation therapy (*p* = 0.248), primary therapy outcome showing PD and SD (*p* = 0.441), male (*p* = 0.284), race belonging to Asian and Black or African American (*p* = 0.477), White race (*p* = 0.059), age of ≤60 years old (*p* = 0.281), lower histologic grades G1 and G2 (*p* = 0.134), higher histologic grades G3 and G4 (*p* = 0.24), being not smoker (*p* = 0.455), without alcohol history (*p* = 0.071), having alcohol history (*p* = 0.306), with lymphovascular invasion (*p* = 0.604), and without lymph node neck dissection (*p* = 0.384).

### 3.10. Results of Survival Analysis by Univariate and Multivariate Cox Regression

Table 4 shows the results of univariate and multivariate cox regression analyses. The univariate analysis results showed that four variables (e.g., radiation therapy, primary therapy outcome, lymphovascular invasion, and DEFB1 expression) were statistically significantly related to the overall survival of OSCC patients, while the other variables (e.g., T stage, N stage, M stage, age, gender, race, smoker, clinical stage, alcohol history, histologic grade, lymph node neck dissection, and anatomic neoplasm subdivision) were not shown to be statistically significantly associated with the overall survival of OSCC patients. The multivariate analysis results showed that several variables (T stage, radiation therapy, primary therapy outcome, lymphovascular invasion, and DEFB1 expression) were statistically significantly associated with the overall survival of OSCC patients; however, the other variables (e.g., N stage, M stage, age, and lymph node neck dissection) were not shown to be associated with the overall survival of OSCC patients.

### 3.11. Forest Plots to Visualize the Results of the Univariate and Multivariate Cox Regression Analyses

Here, one example will be used for interpreting the results of forest plots shown in Figure 3(e): a hazard ratio of 1.424 for DEFB1 low-expression group tells readers that OSCC patients who were detected with the low expression of DEFB1 gene have an increased risk of dying compared to OSCC patients who were detected with the high expression of the DEFB1 gene. The results of univariate Cox regression analysis indicate that several factors (e.g., without receiving radiation therapy (*p* = 0.005), primary therapy outcome of PD and SD (*p* < 0.001), with lymphovascular invasion (*p* = 0.009), and low expression of DEFB1 (*p* = 0.032)) were negative predictors for overall survival outcome in OSCC patients. The results of the multivariate cox regression analysis indicate that several factors (e.g., higher T stage (T3 and T4) (*p* = 0.01), without receiving radiation therapy (*p* = 0.008), primary therapy outcome of PD and SD (*p* < 0.001), with lymphovascular invasion (*p* = 0.021), and low expression of DEFB1 (*p* = 0.024)) were negative predictors for overall survival outcome in OSCC patients. Both univariate and multivariate Cox regression analysis results showed that the DEFB1 expression is an independent prognostic factor correlated with overall survival in OSCC patients.

### 3.12. Nomogram Plot for Risk Estimation

A nomogram plot (Figure 4(a)) was constructed to predict the 1-, 3-, and 5-year survival probability of OSCC patients by integrating the expression level of DEFB1 and independent clinical variables. Total points were calculated by adding the points of the genetic score, age, and TNM stage. A worse prognosis was represented by a higher total number of points on the nomogram.

### 3.13. Calibration Plot for Evaluating the Prediction Accuracy of the Model Established in Nomogram Plot

The calibration curve for predicting 1- and 3-year OS indicated that the nomogram-predicted survival closely corresponded with actual survival outcomes; however, the calibration curve for predicting 5-year OS indicated that the nomogram-predicted survival did not correspond with actual survival outcomes well (Figure 4(b)).

### 3.14. Diagnostic Value of DEFB1 mRNA Expression in OSCC

The diagnostic value of DEFB1 mRNA expression by ROC curve was evaluated.  Figure 5 shows that the predictive ability of DEFB1 gene expression has moderate accuracy in distinguishing the samples of healthy control oral samples versus OSCC tumor samples (AUC = 0.758 (ranging from 0.7 to 0.9), CI = 0.682-0.835). In addition, the diagnostic capability of DEFB1 mRNA expression in predicting different clinical variables was evaluated. Since only two TCGA_OSCC samples were with M1 stage, M stage was not evaluated for the ROC curve analysis. The results showed that the AUC values of all the other clinical variables except for clinical status were less than 0.7 indicating the low diagnostic accuracy (Table 5, Figure 5).

### 3.15. PPI Network Plotting

Figure 6(a) shows that the DEFB1 coexpressed genes constituted the PPI network. Apart from the alpha and beta defensin, DEFB1 was also found to interact with other genes, for instance, BRD4 (Bromodomain Containing 4), BRD2 (Bromodomain Containing 2), and GPR29 (also named CCR6, C-C Motif Chemokine Receptor 6).  Table 6 shows that the representative 10 hub genes were DEFB118, DEFB114, DEFB132, DEFB136, DEFB115, DEFB126, DEFB110, DEFB127, DEFB119, and DEFB113.  Table 6 shows that the most coexpressed genes with DEFB1 were alpha or beta defensin.

### 3.16. GGI Network Plotting

As shown in Figure 6(b), the DEFB1-based GGI network consisted of the DEFB1 gene and its 20 potentially frequently interacting genes and 139 links (interactions). The links included physical interactions (77.64%), coexpression (8.01%), predicated interactions (5.37%), colocalization (3.63%), genetic interactions (2.87%), and pathway (1.88%). The 20 correlated genes of DEFB1 were shown as DEFB103A (defensin beta 103A), CCR6 (C-C motif chemokine receptor 6), MMP7 (matrix metallopeptidase 7), DEFB103B (defensin beta 103B), DEFB130B (defensin beta 130B), DEFB130A (defensin beta 130A), MAP4K2 (mitogen-activated protein kinase kinase kinase kinase 2), SPAG11A (sperm-associated antigen 11A), SPAG11B (sperm-associated antigen 11B), DEFB4A (defensin beta 4A), DEFB4B (defensin beta 4B), FAM172A (family with sequence similarity 172 member A), CCDC198 (coiled-coil domain containing 198), PM20D2 (peptidase M20 domain containing 2), PYROXD2 (pyridine nucleotide-disulphide oxidoreductase domain 2), DDT (D-dopachrome tautomerase), SLC49A3 (solute carrier family 49 member 3), CLDN8 (claudin 8), PTGER3 (prostaglandin E receptor 3), and CXCL1 (C-X-C motif chemokine ligand 1). The functional analysis of the network describes the roles of 21 genes in some biological functions, for example, chemokine receptor binding, CCR chemokine receptor binding, antimicrobial humoral response, G protein-coupled receptor response, humoral immune response, cytokine receptor binding, and positive regulation of cilium movement.

### 3.17. Heatmap Showing the Expression Pattern of Top Correlated Genes of DEFB1 in OSCC

By setting the threshold of ∣cor_pearson | >0.4 and *p*_pearson < 0.001, a total of 549 genes consisting of 69 positively correlated genes and 480 negatively correlated genes were obtained and regarded as the significantly correlated genes of DEFB1. Among these 549 genes, the top 10 positively and top 10 negatively correlated genes were obtained. The top 10 positively correlated genes of DEFB1 were found to be: S100A8 (S100 Calcium Binding Protein A8), S100A9 (S100 Calcium Binding Protein A9), PDZK1IP1 (PDZK1 Interacting Protein 1), SLPI (Secretory Leukocyte Peptidase Inhibitor), BICDL2 (BICD Family Like Cargo Adaptor 2), S100A7 (S100 Calcium Binding Protein A7), SLURP1 (Secreted LY6/PLAUR Domain Containing 1), RASAL1 (RAS Protein Activator Like 1), CAPNS2 (Calpain Small Subunit 2), and RAB25 (Ras-Related Protein Rab-25). The top 10 negatively correlated genes of DEFB1 were found to be EXTL2 (Exostosin-Like Glycosyltransferase 2), AP2B1 (Adaptor-Related Protein Complex 2 Subunit Beta 1), CRTAP (Cartilage-Associated Protein), CNPY4 (Canopy FGF Signaling Regulator 4), XYLT2 (Xylosyltransferase 2), DDOST (Dolichyl-Diphosphooligosaccharide--Protein Glycosyltransferase Non-Catalytic Subunit), AGPAT1 (1-Acylglycerol-3-Phosphate O-Acyltransferase 1), POFUT2 (Protein O-Fucosyltransferase 2), ARMC9 (Armadillo Repeat Containing 9), and BFAR (Bifunctional Apoptosis Regulator).  Figure 6(c) using a heat map shows the expression pattern of these 20 correlated genes in OSCC samples.

### 3.18. Identification of the Biological Functions of the Significantly Correlated Genes of DEFB1

Figure 7(a) uses bubble charts to show the enrichment results in respective to three GO term aspects and KEGG pathways enriched by DEFB1-correlated genes. DEFB1-correlated genes were mainly enriched in several endoplasmic reticulum- (ER-) related biological processes, for example, response to ER stress, protein folding in ER, and ER unfolded protein response. DEFB1-correlated genes were mainly enriched in several ER-related cellular components, for example, ER lumen, ER chaperone complex, ER-Golgi intermediate compartment, integral component of ER membrane, and intrinsic component of ER membrane. DEFB1-correlated genes were mainly enriched in several transferase activity-related molecular functions, for example, fucosyltransferase activity, UDP-glycosyltransferase activity, glucosyltransferase activity, oligosaccharyl transferase activity, UDP-glucosyltransferase activity, UDP-xylosyltransferase activity, and xylosyltransferase activity. Only one KEGG pathway was enriched, which is protein processing in endoplasmic reticulum.

### 3.19. GSEA to Identify the Significant Functional Terms of DEFB1-Correlated Genes

The mountain plot visualized the 17 functional terms according to the criteria of *p*.adjust < 0.05, *q* val < 0.25, and ∣NES | >1 (Figure 7(b)). The enrichment plot showed that DEFB1-significantly correlated genes were mainly enriched in four signaling pathways, ECM (extracellular matrix), RTK/PI3K/AKT/mTOR signaling axis, keratinization, and proinflammatory cytokine-related pathways (Figure 7(b)). Five EMC-related signaling pathways from the Reactome database were significantly enriched, including collagen biosynthesis and modifying enzymes, degradation of the ECM, collagen formation, ECM organization, and vesicle-mediated transport. Five RTK/PI3K/AKT-related pathways from the KEGG database, WP database, and Reactome database were significantly enriched, for instance, focal adhesion, PI3K/AKT/mTOR pathway, PI3K/AKT signaling pathway, and signaling by receptor tyrosine kinases (RTK) which is the upstream pathway of PI3K/AKT signaling axis. Two keratinization-related pathways from the Reactome database were significantly enriched, for instance, formation of the cornified envelope, and keratinization pathway. Two cytokine-related pathways from the WP database were significantly enriched, for instance, VEGFA-VEGFR2 signaling pathway and IL18 signaling pathway.

### 3.20. Identification of the Correlation between DEFB1 Expression and Immune Cells in OSCC

Figure 8(a) (A and B) shows that DEFB1 was significantly positively correlated with several TIICs, including B cells, mast cells, and Th17 cells, while DEFB1 was significantly negatively correlated with several other TIICs, for example, Tgd, macrophages, T helper cells, Tem, Th2 cells, and NK cells. Figure 8(a) (B) shows that the absolute value of the Pearson correlation efficient (*r*) of all TIICs with statistical significance was less than 0.4, indicating the correlation between DEFB1 and immune cells was weak.

### 3.21. Identification of the Correlation between DEFB1 and 15 Typical ICGs

Figure 8(b) (A and B) shows that the DEFB1 expression was significantly correlated with 7 ICGs including HAVCR2, CD276, BTLA, CD70, CD40, TNFSF14, and CD47, while the other ICGs were not found to be statistically correlated with DEFB1 expression. Among these 7 correlated ICGs, only the CD47 gene was positively correlated with DEFB1, while the other 6 genes were found to be negatively correlated with DEFB1 (Figure 8(b) (B)). The absolute value of Pearson correlation efficient (*r*) of these 7 correlated ICGs was less than 0.4, indicating the correlation between DEFB1 expression and these 7 ICGs' expression was weak.

## 4. Discussion

The results of the bioinformatics analyses showed that the DEFB1 regulates tumor biology of OSCC mainly by four signaling pathways, i.e., the extracellular matrix-related pathway, RTK/PI3K/AKT/mTOR pathway, keratinization, and cytokine-related pathway. DEFB1 is involved in the tumor immunity of OSCC by regulating tumor macrophages, mast cells, T cells, and NK cells. In addition, DEFB1 was found strongly correlated with chemokine receptor genes, MAPKs, prostaglandin-related gene, and matrix metallopeptidase family genes. These findings are broadly supported by either direct or indirect experimental evidence.

The current study based on TCGA-OSCC data found a downregulation of DEFB1 in oral cancer samples compared with healthy control samples. In accordance with this finding, a previous study using cell lines found that the mRNA expression level of DEFB1 was significantly lower in oral squamous cell carcinoma cell lines compared with healthy gingival keratinocytes [8]. In addition, the current study showed that a high expression of DEFB1 indicated higher survival probability in terms of overall survival and progress-free survival. Consistent with this finding, a previous study by Han et al. analyzing a cohort of 175 primary OSCC patients found that DEFB1 can be independently regarded as a positive prognostic factor of OSCC, showing that the hBD-1 positive status represented higher cancer-specific survival rate [9]. Furthermore, the current study found that DEFB1 gene expression was not related with lymphovascular invasion; however, it was significantly related with lymph node neck dissection, by showing that DEFB1 expression was significantly lower in the subgroup not receiving dissection surgery compared with the subgroup that received such surgery. To our knowledge, there is only one previous study showing the relationship between DEFB1 expression and lymph node invasion [9]. This study of 175 primary OSCC patients found that DEFB1 expression was significantly lower in OSCC with lymph node metastasis than those without metastasis [9], consistent with our results predicted by computational analysis and thus suggesting that low expression of DEFB1 facilitated the invasion/metastasis of lymph nodes.

The GSEA results showed that DEFB1-significantly correlated genes were mainly enriched in four signaling pathways, ECM (extracellular matrix), RTK/PI3K/AKT/mTOR signaling axis, keratinization, and proinflammatory cytokine-related pathways (e.g., VEGFA-VEGFR2 and IL18). It was found that the expression of matrix metalloproteinase-2 (MMP-2) was downregulated in OSCC cells transfected with DEFB1 compared with OSCC cells without transfection [9]. Matrix metalloproteinases (MMPs) are the main extracellular matrix (ECM) enzymes in collagen degradation; thereby, MMP inhibitors have been considered as a target for anticancer drug agents [27]. These findings indicate an implication of ECM-related signaling pathways in DEFB1-mediated tumor progression. Previous literature investigating nonfunctioning pituitary adenomas has shown that the DEFB1 gene mediated the cytotoxic effect of PI3K/mTOR blockade in pituitary adenomas and in other neuroendocrine tumor cells [28]. The blockade of PI3K/mTOR was found to upregulate the DEFB1 gene, indicating that DEFB1 was a downstream target of the PI3K/mTOR signaling pathway [28]. The increased expression of the DEFB1 gene upon the treatment with PI3K/mTOR inhibitors was found to sensitize the human pancreatic neuroendocrine tumor (NET) cells [28]. The involvement of HBD1 in OSCC has not been reported, but a previous study addressing HBD2 showed a positive expression of HBD2 protein in the keratinized epithelial island of salivary gland tumor [29, 30]. A previous study regarding mBD1 knockout mice found that the knockout of mBD1 was able to trigger the activation of many cytokines, including TGF-*β*, IL-10, IL-1*α*, IL-1*β*, and vascular endothelial growth factor (VEGF) [31]. The mBD1-caused cytokine regulation could lead to the impairment of T cells and NK cells, thereby inducing the further progression of tumors [31].

The current study showed a positive correlation between DEFB1 and B cells and mast cells and a negative correlation between DEFB1 and macrophages and NK cells. The positive correlation between DEFB1 and mast cells seems reasonable since human beta-defensins were found to be able to activate human mast cells and thus induce sustained Ca^2+^ mobilization and substantial degranulation in human mast cells [32]. The degranulation of mast cells activated by DEFB1 was found to prompt the cancer progression by promoting angiogenesis and neovascularization and thus further shaping the tumor microenvironment [33]. In contradiction with the findings predicted by computational biology, an earlier study found a positive correlation between the DEFB1 gene and lymphocytes by showing that the function of lymphocyte T cells was impaired in DEFB1 knockout mice. Previous studies also differ from the findings of this bioinformatics analysis regarding the negative correlation between DEFB1 and macrophages. A previous study showed that the number of tumor-infiltrating macrophages was found to be decreased in mBD1 null tumors of mice [31]. A study regarding another family member of defensins, human beta-defensin 3, showed that hBD-3-expressing tumorigenic cells induced massive tumor infiltration of host macrophages in nude mice, indicating the role of hBD3 in trafficking and recruiting tumor macrophages [34]. Yet, another study regarding beta-defensin 2 showed that vaccination with mBD2 promoted the infiltration of several tumor-infiltrating cells (i.e., CD8+ and CD4+ T, NK cells, and macrophages) in the melanoma tumor tissues [35].

The GGI network showed DEFB1 was correlated with several genes, including CCR6 (C-C motif chemokine receptor 6), CXCL1 (C-X-C motif chemokine ligand 1), MAP4K2 (mitogen-activated protein kinase kinase kinase kinase 2), PTGER3 (prostaglandin E receptor 3), and MMP7 (matrix metallopeptidase 7). There are no reports showing a correlation between human beta-defensin-1 and chemokines or their receptors or ligands; however, other defensin family members, including human beta-defensins 3 and 6, have been found to be associated with chemokines receptors. Previous research regarding human defensin-3 (hBD-3) showed that the chemokine receptor CCR2 played a significant role in recruiting tumor-associated macrophages in response to the exogenous hBD-3 [7, 34]. Another previous research regarding human beta defensin-6 (hBD-6) found that hBD-6 with microvesicles shed by breast cancer cell lines can physically interact with peptides derived from the extracellular domain of CC chemokine receptor 2 (CCR2), indicating that defensins present the chemoattractive activity by interacting with chemokine receptor [36]. Regarding mitogen-activated protein kinase (MAPK) pathway-related molecules, there is no direct evidence showing their correlation with human defensin-1. MAPK molecules have been demonstrated as critical components in regulating the cellular responses to various stimuli, including cytokines and LPS. MAPKs were linked to HBD-2 mRNA expression in epithelial cell-like adenocarcinoma cells—A549 cells [37]. Regarding prostaglandin, previous research by Niyonsaba et al. found that HBD-2 could significantly induce prostaglandin D2 (PGD2) production in mast cells; however, HBD-1 was not observed with such function [38]. The correlation between DEFB1 and MMP7 has been investigated in previous research, and MMP-7-targeted DEFB1 was seen to mediate the generation of amino-terminal variants of HBD-1 [39].

It is worthwhile to highlight the novelty of the present research study investigating the implication of DEFB1 in OSCC. The previous literature mainly provides using molecular cellular experiment data, and such experiments are focused on investigating a selected particular signaling pathway. The current study could identify multiple potentially involved pathways by performing gene correlation analysis and functional enrichment analysis. In addition, individual studies have used small samples to test the gene expression patterns; however, here, we analyzed all samples in TCGA database, providing more robust statistical estimates from a larger sample size. Experimental studies focused to investigate one aspect of gene regulatory role while the current research approach permits investigation of multiple aspects such expression pattern, prognostic values in terms of different survival outcomes, relationship with clinicopathological variables, significantly correlated genes, and potentially involved signaling pathways, as well as the impact on tumor immune cells and immune genes. These comprise the advantages of the present study which can provide meaningful contribution to OSCC research by providing a theoretical basis and experimental direction for future research.

The strengths and limitations of the current research need to be mentioned. This research has used a series of bioinformatics analyses to investigate the implication of the DEFB1 gene in the OSCC tumor comprehensively. The investigated aspects include expression pattern, DNA methylation sites, correlation with clinical variables, prognostic values, significantly correlated genes, involved biological processes and KEGG signaling pathways, and the involvement in tumor immunity. The limitations of the current research chiefly include the lack of experimental validation. Future gene transfection experiments can be designed to address this limitations, and the DEFB1-mediated OSCC mechanisms identified in the current study could be regarded as the theoretical basis of such a research topic and provide experimental directions for future research.

The potential clinical transfer values of the main findings in the current study merit highlighting. Firstly, drug agents targeting DEFB1 have the potential to be an innovative modality for treating oral cancer. The results regarding the subgroup survival analysis (Figure 3(d)) suggest the potential utility of molecular characterization of patient subgroups amenable to therapy with DEFB1 drug targets as a precision medicine approach. DEFB1 represented a prognostic indicator of higher T stage (T3 and T4); thus, using its agonist or modulating its regulated pathway may improve the overall survival outcome of oral cancer patients with higher T stage, while such drug agents may be not meaningful for improving the prognosis in the OSCC patients with lower T stage. Secondly, considering the prognostic value of DEFB1 in OSCC, DEFB1 testing might be meaningful as a prognostic biomarker.

## 5. Conclusion

The downregulation of the DEFB1 gene was found to be a worse prognostic indicator of OSCC. The antitumor role of DEFB1 in OSCC was found to be mainly by four pathways including extracellular matrix-related pathway, RTK/PI3K/AKT/mTOR pathway, keratinization, and cytokines-related pathway. DEFB1 should be regarded as a potential therapeutic target in treating oral cancer.

## Figures and Tables

**Figure 1:** The flowchart showing the study design of the current research.

**Figure 2:** The expression of DEFB1 in pancancer and OSCC. (a) The result of unpaired sample analysis investigating the mRNA levels of six defensin family genes (DEFA1, DEFA3, DEFB1,DEFB103B, DEFB4A, and DEFB114) in OSCC tissues and normal oral tissues in TCGA. (b) The result of paired sample analysis investigating the mRNA levels of six defensin family genes (DEFA1, DEFA3, DEFB1, DEFB103B, DEFB4A, and DEFB114) in OSCC tissues and normal oral tissues in TCGA. (c) The result of unpaired sample analysis investigating the mRNA levels of DEFB1 in OSCC tissues and normal oral tissues in TCGA. (d) The result of paired sample analysis investigating the mRNA levels of DEFB1 in OSCC tissues and normal oral tissues in TCGA. (e) The result of unpaired sample analysis investigating the mRNA expression level of the DEFB1 gene in different tumor types analyzed based on TCGA data. (f) The result of paired sample analysis investigating the mRNA expression level of the DEFB1 gene in different tumor types analyzed based on TCGA data. (g) The correlation between DEFB1 and four methylation sites (cg20710667, cg01691696, cg02465761, and cg24292612). (h) The association of DEFB1 mRNA expression with clinicopathological features, for example, histologic grade (*p* = 0.036), lymph node neck dissection (*p* = 0.014), alcohol history (*p* = 0.006), and OS event (*p* = 0.035).

**Figure 3:** The prognostic value of DEFB1 in OSCC. (a) Survival heat map of hazard ratio (HR) shows the prognostic impacts of the DEFB1 gene on the overall survival (OS) outcomes of multiple cancer types according to the GEPIA2 database. The bounding boxes represented the significant (*p* < 0.05) unfavorable (red) and favorable (blue) results, respectively. (b) Survival heat map of hazard ratio (HR) shows the prognostic impacts of the DEFB1 gene on the disease-free survival (DFS) outcomes of multiple cancer types according to the GEPIA2 database. (c) The prognostic values of DEFB1 in OSCC from the aspect of three types of prognostic parameters (i.e., overall survival, disease-specific survival, and progress-free interval). (d) The subgroup survival analysis showing the association between DEFB1 mRNA overexpression and overall survival outcome of OSCC in specific subgroups dividing by the clinical characteristics, for example, higher T stage T3 and T4; M stage M0; gender: female; age: >60; smoker: yes; radiation therapy: no; primary therapy outcome: PR and CR; lymphovascular invasion: no; and lymph node dissection: yes. (e) The forest plots showing the univariate and multivariate regression analysis results of DEFB1 and clinicopathologic parameters with overall survival (OS) in OSCC patients.

**Figure 4:** Nomogram plot and calibration plot. (a) Nomogram plot for predicting probability of patients with 1-, 3-, and 5-year overall survival. (b) Calibration curve for nomogram-predicted 1-year, 3-year, and 5-year overall survival. The *x*-axis is the nomogram-predicted survival probability, and the *y*-axis is the observed survival probability, respectively.

**Figure 5:** The ROC curves evaluating the diagnostic values of the DEFB1 gene in predicting a variety of clinicopathologic variables including clinical status (tumor vs. control), T stage (T3 and T4 vs. T1 and T2), N stage (N1 and N2 and N3 vs. N0), clinical stage (Stages III and IV vs. Stages I and II), histologic grade (G3 and G4 vs. G1 and G2), radiation therapy (no vs. yes), primary therapy outcome \n (PD and SD vs. PR and CR), gender (male vs. female), race (Asian and Black vs. White), age (>60 vs. <60), smoker (yes vs. no), alcohol history (yes vs. no), lymphovascular invasion (yes vs. no), lymph node neck dissection (no vs. yes), OS events (dead vs. alive), DSS events (dead vs. alive), and PFI events (dead vs. alive).

**Figure 6:** The DEFB1-correlated genes. (a) The DEFB1 coexpressed genes constituted the protein-protein interaction network, which was constructed by STRING software. (b) The gene-gene interaction networks designed by using GeneMania webserver. (c) Heatmap showing the expression pattern of the top 10 positively and negatively correlated genes in OSCC samples.

**Figure 7:** The biological functions enriched by DEFB1-correlated genes. (a) The functional enrichment analysis results of the significantly correlated genes of DEFB1, in terms of GO terms—BP (biological process); CC (cellular component); MF (molecular function); and KEGG pathways. (b) The results obtained by GSEA, which were visualized by mountain plot and enrichment plot. The mountain plot showed the functional terms obtained by GSEA, according to the criteria of *p*.adjust < 0.05, *q* val < 0.25, and ∣NES | >1. The enrichment plot showed that DEFB1-significantly correlated genes were mainly enriched in four signaling pathways, ECM (extracellular matrix), RTK (receptor tyrosine kinases)/PI3K/AKT signaling axis, keratinization, and proinflammatory cytokine-related pathways.

**Figure 8:** The involvement of the DEFB1 gene in tumor immunity of OSCC. (a) Results regarding the correlation between DEFB1 expression and tumor immune infiltrating cells. (A) Lollipop plot showing the correlation between DEFB1 expression and 24 TIICs in OSCC. (B) Scatter plots showing the significant positive correlation between DEFB1 expression and 3 types of TIICs (i.e., B cells, mast cells, and Th17 cells) and the significant negative correlation between DEFB1 expression and 6 types of TIICs (i.e., Tgd, macrophages, T helper cells, Tem, Th2 cells, and NK cells). (b) Results regarding the correlation between DEFB1 expression and 15 ICGs in OSCC tumor samples. (A) The heat map showing the expression pattern of 15 ICGs in OSCC; (B) scatter plots showing the statistically significant correlation between DEFB1 expression and several genes (HAVCR2, CD276, BTLA, CD70, CD40, CD47, and TNFSF14).

**Table 1:** The ADP ID, source, and encoded genes of 23 oral-sourced human ADMs obtained from the ADP database.

APD ID	Name	Source	Gene symbol
AP00176	Human neutrophil peptide-1 (HNP-1, HNP1, alpha Defensin, UCSS1a; lectin; primates, mammals, animals; XXX; ZZHh, BBS; BBL; BBW; 3S=S)	Neutrophils; natural killer cells, monocytes; saliva; Homo sapiens	DEFA1
AP00177	Human neutrophil peptide-2 (HNP-2, HNP2, alpha Defensin, lectin; UCSS1a; primates, mammals, animals; ZZHh, BBS; 3S=S; BBMm)	Neutrophils; natural killer cells, monocytes; saliva; Homo sapiens	DEFA1
AP00178	Human neutrophil peptide-3 (HNP-3, HNP3, alpha Defensin, UCSS1a; primates, mammals, animals; lectin; ZZHh, BBS; 3S=S)	Neutrophils; natural killer cells, monocytes; saliva; Homo sapiens	DEFA3
AP00451	hBD-1 (human beta-defensin 1; hBD1; 3S=S; UCSS1a; primates, mammals, animals; ZZH, JJsn; XXR)	Hemofiltrates, urine, kidney; keratinocytes; skin; platelets; oral saliva; milk, mammary gland epithelium, Homo sapiens	DEFB1
AP00524	Human beta defensin 2 (hBD-2; hBD2; UCSS1a; human, primates, mammals, animals; ZZHh; 3S=S; JJsn)	Skin, lung, trachea epithelia, and uterus, oral (saliva); Homo sapiens	DEFB4A
AP00283	Human beta defensin 3 (hBD-3, hBD3, or DEFB103, human defensin, 3S=S, UCSS1a; primates, mammals, animals; ZZHh; BBBh2o; BBW; JJsn)	Skin, tonsils, oral/saliva, Homo sapiens	DEFB103B
AP02182	DEFB114 (human beta defensin 114, UCSS1a; 4S=S, primates, mammals, animals; BBL)	Epididymis and gingival cells, Homo sapiens	DEFB114
AP00798	Human Histatin 1 (XXP) (Hst1; His-rich; primates, mammals, animals)	Human saliva, Homo sapiens	HTN1
AP00799	Human Histatin 2 (His-rich; primates, mammals, animals)	Human saliva, Homo sapiens	HTN3
AP00520	Human Histatin 3 (His-rich, primates, mammals, animals; BBII)	Saliva; Homo sapiens	HTN3
AP00800	Human Histatin 4 (His-rich; primates, mammals, animals)	Human saliva, Homo sapiens	HTN3
AP00505	Human Histatin 5 (hst5; primates, mammals, animals; His-rich; ZZHs; BBII; derivatives: Dh-5; Dhvar5; Dhvar4; demegen P-113; P113; clinical)	Salivary glands, Homo sapiens	HTN3
AP00801	Human Histatin 6 (His-rich; primates, mammals, animals)	Human saliva, Homo sapiens	HTN3
AP00802	Human Histatin 7 (His-rich; primates, mammals, animals)	Human saliva, Homo sapiens	HTN3
AP00803	Human histatin 9 (His-rich; primates, mammals, animals. Other derivatives detected are Histatin 10, Histatin 11, and Histatin 12)	Human saliva, Homo sapiens	HTN3
AP00310	LL-37 [LL37; FALL-39; cathelicidin; UCLL1; human; chimpanzee; primates, mammals, animals; XXX; XXY; XXZ; BBBh2o, BBBm; BBMm, BBPP, BBN, BBL, BBrsg, JJsn; derivatives: many)	Neutrophils, monocytes; mast cells; lymphocytes, mesenchymal stem cells; islets; skin, sweat; airway surface liquid, saliva; Homo sapiens; also Pan troglodytes	CAMP
AP00765	Human salvic (primates, mammals, animals)	Salivary gland, Homo sapiens	C77-91 (not included in GeneCards database)
AP01479	Adrenomedullin (AM; ADM; neuropeptide; hypotensitve peptide; 1S=S; UCSS1a; human; primates, mammals, animals; XXA)	Adrenal medulla, skin, oral/saliva; Homo sapiens	ADM
AP02072	Psoriasin (S100A7; metal-binding protein, BBII; humans; primates, mammals, animals)	Keratinocytes, skin (e.g., hair follicle), tongue Homo sapiens	S100A7
AP02095	SLPI (secretory leukocyte protease inhibitor, antileukoprotease, ALP, UCSS1a; human, primates, mammals, animals; 8S=S; BBMm; BBN)	Tears, saliva, airway, gastrointestines, genital tracts, Homo sapiens	SLPI
AP02186	CCL28 (MEC; SCYA28; CCK1; cytokine, kinocidins; human, primates, mammals, animals)	Saliva, milk, epithelial cells/mucosal tissues, Homo sapiens	CCL28
AP02257	Lysozyme (lectin-binding enzyme, human, primates, mammals, animals; BBS; JJsn; UCSS1a)	Secretions and tissues, tears, saliva, human milk, and mucus; Homo sapiens	LYZ
AP02519	sfTSLP (short-form thymic stromal lymphopoietin, isoform 2, cytokine, human, primates, mammals, animals; other fragments: MKK34)	Keratinocytes, oral mucosa/salivary glands, skin, gut, Homo sapiens	TSLP

**Table 2:** The clinical characteristics of the TCGA-OSCC patients depending on the expression level of DEFB1 gene.

Characteristic	Levels	Low expression of DEFB1	High expression of DEFB1	*p*
*n*		164	165	
T stage, *n* (%)	T1	10 (3.1%)	8 (2.5%)	0.964
	T2	53 (16.6%)	52 (16.3%)	
	T3	40 (12.5%)	42 (13.2%)	
	T4	57 (17.9%)	57 (17.9%)	
N stage, *n* (%)	N0	78 (24.8%)	90 (28.6%)	0.415
	N1	31 (9.8%)	25 (7.9%)	
	N2	49 (15.6%)	39 (12.4%)	
	N3	1 (0.3%)	2 (0.6%)	
M stage, *n* (%)	M0	156 (50%)	154 (49.4%)	1.000
	M1	1 (0.3%)	1 (0.3%)	
Clinical stage, *n* (%)	Stage I	6 (1.9%)	5 (1.6%)	0.887
	Stage II	37 (11.6%)	42 (13.2%)	
	Stage III	32 (10%)	33 (10.3%)	
	Stage IV	85 (26.6%)	79 (24.8%)	
Radiation therapy, *n* (%)	No	60 (20.3%)	56 (19%)	0.828
	Yes	89 (30.2%)	90 (30.5%)	
Primary therapy outcome, *n* (%)	PD	16 (5.8%)	19 (6.8%)	0.312
	SD	3 (1.1%)	1 (0.4%)	
	PR	3 (1.1%)	0 (0%)	
	CR	121 (43.5%)	115 (41.4%)	
Gender, *n* (%)	Female	49 (14.9%)	53 (16.1%)	0.748
	Male	115 (35%)	112 (34%)	
Race, *n* (%)	Asian	3 (0.9%)	6 (1.9%)	0.684
	Black or African American	11 (3.5%)	10 (3.1%)	
	White	144 (45.3%)	144 (45.3%)	
Age, *n* (%)	≤60	81 (24.7%)	74 (22.6%)	0.442
	>60	82 (25%)	91 (27.7%)	
Histologic grade, *n* (%)	G1	17 (5.3%)	35 (10.9%)	0.043
	G2	105 (32.7%)	95 (29.6%)	
	G3	36 (11.2%)	31 (9.7%)	
	G4	1 (0.3%)	1 (0.3%)	
Anatomic neoplasm subdivision, *n* (%)	Alveolar ridge	6 (1.8%)	12 (3.6%)	0.250
	Base of tongue	12 (3.6%)	11 (3.3%)	
	Buccal mucosa	14 (4.3%)	8 (2.4%)	
	Floor of mouth	33 (10%)	28 (8.5%)	
	Hard palate	1 (0.3%)	6 (1.8%)	
	Oral cavity	37 (11.2%)	35 (10.6%)	
	Oral tongue	61 (18.5%)	65 (19.8%)	
Smoker, *n* (%)	No	43 (13.3%)	44 (13.6%)	1.000
	Yes	118 (36.5%)	118 (36.5%)	
Alcohol history, *n* (%)	No	41 (12.8%)	64 (19.9%)	0.012
	Yes	118 (36.8%)	98 (30.5%)	
Lymphovascular invasion, *n* (%)	No	81 (33.9%)	83 (34.7%)	0.965
	Yes	38 (15.9%)	37 (15.5%)	
Lymph node neck dissection, *n* (%)	No	28 (8.6%)	17 (5.2%)	0.104
	Yes	135 (41.3%)	147 (45%)	
OS event, *n* (%)	Alive	82 (24.9%)	97 (29.5%)	0.136
	Dead	82 (24.9%)	68 (20.7%)	
DSS event, *n* (%)	Alive	105 (33.7%)	114 (36.5%)	0.414
	Dead	50 (16%)	43 (13.8%)	
PFI event, *n* (%)	Alive	90 (27.4%)	104 (31.6%)	0.164
	Dead	74 (22.5%)	61 (18.5%)	
Age, median (IQR)		61 (52, 71)	62 (55, 69)	0.524

**Table 3:** Logistic regression analysis results showing the association between DEFB1 expression and clinical characteristics.

Characteristics	Total (*N*)	Odds ratio (OR) (95% confidence interval (CI))	*p* value
T stage (T3 & T4 vs. T1 & T2)	319	1.072 (0.682-1.684)	0.764
N stage (N1 & N2 & N3 vs. N0)	315	0.706 (0.452-1.100)	0.125
M stage (M1 vs. M0)	312	1.013 (0.040-25.769)	0.993
Clinical stage (Stage III & Stage IV vs. Stage I & Stage II)	319	0.876 (0.537-1.427)	0.594
Histologic grade (G3 & G4 vs. G1 & G2)	321	0.812 (0.474-1.383)	0.443
Gender (male vs. female)	329	0.900 (0.563-1.437)	0.660
Race (Asian & Black or African American vs. White)	318	1.143 (0.537-2.457)	0.728
Age (>60 vs. ≤60)	328	1.215 (0.787-1.877)	0.380
Smoker (yes vs. no)	323	0.977 (0.597-1.599)	0.927
Alcohol history (yes vs. no)	321	0.532 (0.329-0.853)	0.009
Primary therapy outcome (PD & SD vs. PR & CR)	278	1.135 (0.575-2.247)	0.714
Radiation therapy (no vs. yes)	295	0.923 (0.578-1.473)	0.737
Lymph node neck dissection (no vs. yes)	327	0.558 (0.287-1.054)	0.076
Lymphovascular invasion (yes vs. no)	239	0.950 (0.549-1.643)	0.855
Anatomic neoplasm subdivision (oral cavity & hard palate & floor of mouth & buccal mucosa & base of tongue & alveolar ridge vs. oral tongue)	329	0.911 (0.583-1.422)	0.682

**Table 4:** The correlations between overall survival and mRNA expression of DEFB1 analyzed by univariate and multivariate Cox regression.

Characteristics	Total (*N*)	Univariate analysis		Multivariate analysis	
		HR (95% CI)	*p* value	HR (95% CI)	*p* value
T stage (T3 & T4 vs. T1 & T2)	318	1.363 (0.971-1.913)	0.074	2.111 (1.195-3.730)	0.010
N stage (N1 & N2 & N3 vs. N0)	314	1.320 (0.955-1.824)	0.092	1.321 (0.800-2.183)	0.277
M stage (M1 vs. M0)	311	2.621 (0.365-18.838)	0.338		
Age (>60 vs. ≤60)	328	1.320 (0.954-1.826)	0.094	1.058 (0.658-1.702)	0.816
Gender (male vs. female)	328	0.908 (0.648-1.273)	0.576		
Race (Asian & Black or African American vs. White)	318	1.532 (0.880-2.667)	0.131		
Smoker (yes vs. no)	322	1.248 (0.845-1.844)	0.265		
Clinical stage (Stage III & Stage IV vs. Stage I & Stage II)	318	1.282 (0.889-1.848)	0.183		
Alcohol history (yes vs. no)	320	1.045 (0.740-1.475)	0.804		
Histologic grade (G3 & G4 vs. G1 & G2)	320	1.252 (0.862-1.820)	0.238		
Radiation therapy (no. vs. yes)	294	1.663 (1.164-2.377)	0.005	2.012 (1.195-3.385)	0.008
Primary therapy outcome (PD & SD vs. PR & CR)	277	5.472 (3.540-8.457)	<0.001	3.647 (2.174-6.119)	<0.001
Lymphovascular invasion (yes vs. no)	238	1.698 (1.141-2.529)	0.009	1.788 (1.091-2.930)	0.021
Lymph node neck dissection (no. vs. yes)	326	1.462 (0.964-2.216)	0.074	2.004 (0.847-4.742)	0.114
Anatomic neoplasm subdivision (floor of mouth vs. oral tongue)	186	1.471 (0.937-2.307)	0.093		
Anatomic neoplasm subdivision (oral cavity vs. oral tongue)	197	1.161 (0.766-1.761)	0.482		
Anatomic neoplasm subdivision (base of tongue vs. oral tongue)	148	1.004 (0.493-2.048)	0.990		
Anatomic neoplasm subdivision (buccal mucosa vs. oral tongue)	147	0.965 (0.474-1.965)	0.922		
Anatomic neoplasm subdivision (alveolar ridge vs. oral tongue)	143	0.870 (0.394-1.921)	0.730		
DEFB1 expression (low vs. high)	328	1.424 (1.031-1.967)	0.032	1.694 (1.072-2.679)	0.024

**Table 5:** The parameters of the all predicted outcomes in ROC curves. These parameters include area under the curves (AUC), confidence interval (CI), cutoff value, sensitivity, specificity, positive predictive value, negative predictive value, and Youden index.

Predicted outcomes	AUC	CI	Cutoff value	Sensitivity	Specificity	Positive predictive value	Negative predictive value	Youden index
Clinical status (tumor vs. normal)	0.758	0.682-0.835	7.08	0.626	0.844	0.976	0.18	0.47
T stage (T3 & T4 vs. T1 & T2)	0.499	0.434-0.564	8.079	0.214	0.829	0.667	0.398	0.044
N stage (N1 & N2 & N3 vs. N0)	0.559	0.495-0.623	6.018	0.483	0.667	0.559	0.596	0.15
Clinical stage (Stage III & Stage IV vs. Stage I & Stage II)	0.534	0.466-0.603	5.631	0.367	0.778	0.808	0.326	0.145
Histologic grade (G3 & G4 vs. G1 & G2)	0.566	0.483-0.648	4.915	0.333	0.849	0.377	0.823	0.183
Gender (male vs. female)	0.544	0.477-0.610	4.154	0.194	0.931	0.863	0.342	0.125
Race (Asian & Black or African American vs. White)	0.498	0.394-0.602	6.712	0.533	0.552	0.11	0.919	0.085
Age (>60 vs. ≤60)	0.536	0.473-0.599	7.42	0.341	0.755	0.608	0.506	0.096
Smoker (yes vs. no)	0.471	0.401-0.541	9.097	0.072	0.943	0.773	0.272	0.015
Alcohol history (yes vs. no)	0.595	0.529-0.661	7.046	0.681	0.524	0.746	0.444	0.204
Anatomic neoplasm (alveolar ridge & base of tongue & buccal mucosa & floor of mouth & hard palate & oral cavity vs. oral tongue)	0.524	0.460-0.588	5.706	0.374	0.714	0.679	0.415	0.089
Primary therapy outcome (PD & SD vs. PR & CR)	0.525	0.421-0.629	7.428	0.385	0.728	0.188	0.879	0.113
Radiation therapy (no. vs. yes)	0.478	0.411-0.546	6.754	0.578	0.453	0.406	0.623	0.03
Lymphovascular invasion (yes vs. no)	0.54	0.462-0.619	7.712	0.84	0.274	0.346	0.789	0.114
Lymph node neck dissection (no vs. yes)	0.614	0.523-0.706	5.763	0.533	0.677	0.209	0.901	0.211
OS (overall survival) event (dead vs. alive)	0.567	0.505-0.630	6.862	0.647	0.486	0.513	0.621	0.133
DSS (disease-specific survival) event (dead vs. alive)	0.546	0.476-0.616	5.025	0.28	0.822	0.4	0.729	0.101
PFI (progression-free survival) event (dead vs. alive)	0.545	0.481-0.608	6.826	0.63	0.479	0.457	0.65	0.109

**Table 6:** The correlations between the representative 10 hub genes with DEFB1 in OSCC patients.

Name	Description	Degree	*r* (correlation coefficient)
DEFB118	Defensin beta 118	30	-0.012039552
DEFB114	Defensin beta 114	30	-0.017218944
DEFB132	Defensin beta 110	30	-0.052537384
DEFB136	Defensin beta 136	30	-0.027379147
DEFB115	Defensin beta 115	30	0.094748542
DEFB126	Defensin beta 126	30	0.027400918
DEFB110	Defensin beta 110	30	0.081281382
DEFB127	Defensin beta 127	30	0.111490401
DEFB119	Defensin beta 119	30	-0.115552915
DEFB113	Defensin beta 113	30	0.021481822

## Data Availability

The data analyzed during the current study are available in TCGA database with the accession numbers TCGA-HNSC. The original contributions presented in the study are included in the article; further inquiries can be directed to the two equally corresponding authors.

## References

[1] Lei J., Sun L., Huang S. (2019). The antimicrobial peptides and their potential clinical applications. *American Journal of Translational Research*.

[2] Sun Y., Shang D. (2015). Inhibitory effects of antimicrobial peptides on lipopolysaccharide-induced inflammation. *Mediators of Inflammation*.

[3] Diamond G., Beckloff N., Weinberg A., Kisich K. O. (2009). The roles of antimicrobial peptides in innate host defense. *Current Pharmaceutical Design*.

[4] Hoskin D. W., Ramamoorthy A. (2008). Studies on anticancer activities of antimicrobial peptides. *Biochimica et Biophysica Acta*.

[5] Xu D., Lu W. (2020). Defensins: a double-edged sword in host immunity. *Frontiers in Immunology*.

[6] Wang Z., Wang G. (2004). APD: the antimicrobial peptide database. *Nucleic Acids Research*.

[7] Ghosh S. K., McCormick T. S., Weinberg A. (2019). Human beta defensins and cancer: contradictions and common ground. *Frontiers in Oncology*.

[8] Joly S., Compton L. M., Pujol C., Kurago Z. B., Guthmiller J. M. (2009). Loss of human beta-defensin 1, 2, and 3 expression in oral squamous cell carcinoma. *Oral Microbiology and Immunology*.

[9] Han Q., Wang R., Sun C. (2014). Human beta-defensin-1 suppresses tumor migration and invasion and is an independent predictor for survival of oral squamous cell carcinoma patients. *PLoS One*.

[10] Vivian J., Rao A. A., Nothaft F. A. (2017). Toil enables reproducible, open source, big biomedical data analyses. *Nature Biotechnology*.

[11] Modhukur V., Iljasenko T., Metsalu T., Lokk K., Laisk-Podar T., Vilo J. (2018). MethSurv: a web tool to perform multivariable survival analysis using DNA methylation data. *Epigenomics*.

[12] Tang Z., Li C., Kang B., Gao G., Li C., Zhang Z. (2017). GEPIA: a web server for cancer and normal gene expression profiling and interactive analyses. *Nucleic Acids Research*.

[13] Love M. I., Huber W., Anders S. (2014). Moderated estimation of fold change and dispersion for RNA-seq data with DESeq2. *Genome Biology*.

[14] Subramanian A., Tamayo P., Mootha V. K. (2005). Gene set enrichment analysis: a knowledge-based approach for interpreting genome-wide expression profiles. *Proceedings of the National Academy of Sciences of the United States of America*.

[15] Yu G., Wang L. G., Han Y., He Q. Y. (2012). clusterProfiler: an R package for comparing biological themes among gene clusters. *OMICS*.

[16] Hänzelmann S., Castelo R., Guinney J. (2013). GSVA: gene set variation analysis for microarray and RNA-seq data. *BMC Bioinformatics*.

[17] Bindea G., Mlecnik B., Tosolini M. (2013). Spatiotemporal dynamics of intratumoral immune cells reveal the immune landscape in human cancer. *Immunity*.

[18] Veigas F., Mahmoud Y. D., Merlo J., Rinflerch A., Rabinovich G. A., Girotti M. R. (2021). Immune checkpoints pathways in head and neck squamous cell carcinoma. *Cancers (Basel)*.

[19] Jia Y. Q., Yang B., Wen L. L., Mu W. X., Wang Z., Cheng B. (2019). Prognostic value of immune checkpoint molecules in head and neck cancer: a meta-analysis. *Aging (Albany NY)*.

[20] Zhu L., Ma N., Wang B. (2019). Significant prognostic values of aquaporin mRNA expression in breast cancer. *Cancer Management and Research*.

[21] Yu S., Wu Y., Li C. (2020). Comprehensive analysis of the SLC16A gene family in pancreatic cancer via integrated bioinformatics. *Scientific Reports*.

[22] Li Z., Liu Z., Shao Z. (2020). Identifying multiple collagen gene family members as potential gastric cancer biomarkers using integrated bioinformatics analysis. *PeerJ*.

[23] Zeng M.-L., Zhu X.-J., Liu J. (2020). An integrated bioinformatic analysis of the S100 gene family for the prognosis of colorectal cancer. *BioMed Research International*.

[24] Xu S., Wang Y., Li Y., Zhang L., Wang C., Wu X. (2020). Comprehensive analysis of inhibitor of differentiation/DNA-binding gene family in lung cancer using bioinformatics methods. *Bioscience Reports*.

[25] Hu Y., Zheng M., Zhang D. (2021). Identification of the prognostic value of a 2-gene signature of the WNT gene family in UCEC using bioinformatics and real-world data. *Cancer Cell International*.

[26] Wang L., Xu D., Cai L., Dai J., Li Y., Xu H. (2021). Expression and survival analysis of the STAT gene family in diffuse gliomas using integrated bioinformatics. *Current Research in Translational Medicine*.

[27] Jabłońska-Trypuć A., Matejczyk M., Rosochacki S. (2016). Matrix metalloproteinases (MMPs), the main extracellular matrix (ECM) enzymes in collagen degradation, as a target for anticancer drugs. *Journal of Enzyme Inhibition and Medicinal Chemistry*.

[28] Lee M., Wiedemann T., Gross C. (2015). Targeting PI3K/mTOR signaling displays potent antitumor efficacy against nonfunctioning pituitary adenomas. *Clinical Cancer Research*.

[29] Abiko Y., Nishimura M., Kusano K., Kaku T. (2000). Presence of human beta-defensin 2 peptide in keratinization in salivary gland tumor. *Oral Medicine & Pathology*.

[30] Abiko Y., Suraweera A. K., Nishimura M. (2001). Differential expression of human beta-defensin 2 in keratinized and non-keratinized oral epithelial lesions; immunohistochemistry and in situ hybridization. *Virchows Archiv*.

[31] Sun C. Q., Arnold R. S., Hsieh C. L. (2019). Discovery and mechanisms of host defense to oncogenesis: targeting the *β*-defensin-1 peptide as a natural tumor inhibitor. *Cancer Biology & Therapy*.

[32] Agier J., Brzezińska-Błaszczyk E., Różalska S., Wiktorska M., Wawrocki S., Żelechowska P. (2020). *β*-Defensin strengthens antimicrobial peritoneal mast cell response. *Journal of Immunology Research*.

[33] Komi D. E. A., Redegeld F. A. (2020). Role of mast cells in shaping the tumor microenvironment. *Clinical Reviews in Allergy & Immunology*.

[34] Jin G., Kawsar H. I., Hirsch S. A. (2010). An antimicrobial peptide regulates tumor-associated macrophage trafficking via the chemokine receptor CCR2, a model for tumorigenesis. *PLoS One*.

[35] Mei H.-f., Jin X.-b., Zhu J.-y. (2012). *β*-Defensin 2 as an adjuvant promotes anti-melanoma immune responses and inhibits the growth of implanted murine melanoma in vivo. *PloS One*.

[36] de Paula V. S., Gomes N., Lima L. (2013). Structural basis for the interaction of human *β*-defensin 6 and its putative chemokine receptor CCR2 and breast cancer microvesicles. *Journal of Molecular Biology*.

[37] Jang B.-C., Lim K.-J., Suh M.-H., Park J.-G., Suh S.-I. (2007). Dexamethasone suppresses interleukin-1Î²-induced human Î²-defensin 2 mRNA expression: involvement of p38 MAPK, JNK, MKP-1, and NF-ÎºB transcriptional factor in A549 cells. *FEMS Immunology & Medical Microbiology*.

[38] Niyonsaba F., Someya A., Hirata M., Ogawa H., Nagaoka I. (2001). Evaluation of the effects of peptide antibiotics human beta-defensins-1/-2 and LL-37 on histamine release and prostaglandin D_2_ production from mast cells. *European Journal of Immunology*.

[39] Wilson C. L., Schmidt A. P., Pirilä E. (2009). Differential processing of *α*- and *β*-defensin precursors by matrix metalloproteinase-7 (MMP-7). *The Journal of Biological Chemistry*.

